# Identification of Tumor Tissue of Origin with RNA-Seq Data and Using Gradient Boosting Strategy

This article has been retracted.

**DOI:** 10.1155/2021/6653793

**Published:** 2021-02-17

**Authors:** Ruixi Li, Bo Liao, Bo Wang, Chan Dai, Xin Liang, Geng Tian, Fangxiang Wu

**Affiliations:** ^1^School of Mathematics and Statistics, Hainan Normal University, Haikou 570100, China; ^2^Key Laboratory of Computational Science and Application of Hainan Province, Haikou 571158, China; ^3^Key Laboratory of Data Science and Intelligence Education (Hainan Normal University), Ministry of Education, Haikou 571158, China; ^4^Qingdao Geneis Institute of Big Data Mining and Precision Medicine, Qingdao 266000, China; ^5^Geneis (Beijing) Co., Ltd., Beijing 100102, China; ^6^Division of Biomedical Engineering, Department of Mechanical Engineering, University of Saskatchewan, Saskatoon, SK, S7N5A9, Canada

## Abstract

**Background:**

Cancer of unknown primary (CUP) is a type of malignant tumor, which is histologically diagnosed as a metastatic carcinoma while the tissue-of-origin cannot be identified. CUP accounts for roughly 5% of all cancers. Traditional treatment for CUP is primarily broad-spectrum chemotherapy; however, the prognosis is relatively poor. Thus, it is of clinical importance to accurately infer the tissue-of-origin of CUP.

**Methods:**

We developed a gradient boosting framework to trace tissue-of-origin of 20 types of solid tumors. Specifically, we downloaded the expression profiles of 20,501 genes for 7713 samples from The Cancer Genome Atlas (TCGA), which were used as the training data set. The RNA-seq data of 79 tumor samples from 6 cancer types with known origins were also downloaded from the Gene Expression Omnibus (GEO) for an independent data set.

**Results:**

400 genes were selected to train a gradient boosting model for identification of the primary site of the tumor. The overall 10-fold cross-validation accuracy of our method was 96.1% across 20 types of cancer, while the accuracy for the independent data set reached 83.5%.

**Conclusion:**

Our gradient boosting framework was proven to be accurate in identifying tumor tissue-of-origin on both training data and independent testing data, which might be of practical usage.

## 1. Introduction

Cancer of unknown primary (CUP) is a type of malignant tumor, histologically diagnosed as a metastatic carcinoma with no confidently anatomical primary site even after comprehensive evaluation. CUP accounts for approximately 3% to 5% of all tumors [1–4]. In general, primary cancer tissue can be identified at the same time as diagnosis. However, for some patients, it is relatively difficult to identify cancer tissue-of-origin since the markers for origin tracing is unidentifiable. Previous studies showed that less than 50% of CUPs could be accurately diagnosed [5–8]. Accurate classification of the tumor types according to anatomical and histological assays is urgent [9–11].

The patients diagnosed as CUP are treated by using traditional chemotherapy; however, prognoses of these patients are relatively poor. For a physician, accurate diagnosis can be a direct guide to individual surgical intervention as well as medication regimen. Furthermore, identification of the primary site of the tumor is relatively helpful for clinicians to design a targeted treatment plan, as well as improving survivals and quality of life [12, 13].

Currently, the diagnostic techniques primarily include comprehensive evaluation, imaging examination, pathological analysis, immunohistochemistry (IHC) panels, and genetic testing [2]. A gene expression-based test is considered as an adjunct test to an uncertain diagnosis of biopsy; moreover, it provides a new approach for the cancer diagnosis of predicting the prognosis of tumors [12]. Many cancerous cells retain features of their primary tissues of origin during metastasis; in other words, gene expression of metastatic cancer should be consistent with the gene expression of its primary tissue [14, 15]. It has been found that the gene expression profiles of metastatic tumors were different from the tissue of the metastatic site but more similar to those at the primary origin. A gene expression profile of the tissue origin is always retained during the process of tumor occurrence, development, and metastasis. Based on this theory, researchers developed a series of molecular markers of gene expression to trace the tissue origin of tumors.

CancerTYPE ID was a gene expression-based test, focusing on identifying the tissue of origin. This molecular test was based on real-time PCR technology by using the differential expression data of 92 genes in the tumor cells and classified tumors by matching the gene expression partem of tumor specimens to a database of 50 known tumor types and subtypes. The test compared genomic information from tumor samples with reference databases of more than 2000 tumors with definitive diagnoses. Gene expression profile analysis by using microarray data provided diagnoses of cancer types with high accuracy [7]. Another gene expression-based test named the Pathwork Tissue of Origin (TOO) test also contributes to improve the diagnosis of CUP. The Pathwork Tissue of Origin test applied a microarray-based expression profile of 2000 gene markers to assess the molecular similarity of the patient tumor with a panel of 15 known Genomic Test for Tumor Origin in formalin-fixed, paraffin-embedded (FFPE) tissues. This method primarily included two algorithms, one for standardization and the other for classification [2, 16].

RNA-seq is a high-throughput sequencing approach that sequences mRNA, small RNA, and noncoding RNA by using high-throughput sequencing technology. RNA-seq, characterized with more exact quantification, higher repeatability, wider examination area, and more credible analysis, can be used to study genome-wide differences in gene expression. In addition, it is considered as cost-effective. TOO was based on Array data, and CancerTYPE ID was conducted on the RT-PCR data; however, application of RT-PCR or Array has not only a higher cost but also a limited accuracy. Here, we conducted an experiment to identify the tissue of origin with a gradient boosting classifier [17] and RNA-seq technique.

## 2. Materials and Methods

### 2.1. Data Preparation

The Cancer Genome Atlas (TCGA) RNA-seq and array data include 20,501 genes from the ICGC Data Portal (https://dcc.icgc.org/releases/release_26/) download. In order to facilitate the follow-up work, we generated a *M*∗*N* matrix where *M* represents the sample size and *N* represents the number of genes. The matrix was generated by normalizing the expression value of each sample and each gene from TCGA. An independent data set, including 79 tumor samples from 6 cancer types with known origins, was also downloaded from the Gene Expression Omnibus (GEO). These samples belong to GSE8352, GSE8734, GSE11107, GSE11132, GSE4895, GSE6491, GSE7966, GSE7766, and GSE11843. The samples not included in the 20 cancers were excluded.

### 2.2. Gene Selection and Classification

We employed a gradient boosting algorithm for gene feature selection and final classification with cross-validation. Gradient boosting (GBDT) is a machine learning method for regression and classification in studies, which combines multiple weak learners into prediction models [18]. Furthermore, the weak learner is usually a decision tree. In the GBDT iteration, we assume that the strong learner obtained in the previous iteration is *f*_*t*−1_(*x*) and the loss function is *L*(*y*, *f*_*t*‐1_(*x*)). The goal of this round of iterations is to find a weak-learner *h*_*t*_(*x*) of the CART regression tree model and minimize the loss function *L*(*y*, *f*_*t*_(*x*) = *f*_*t*‐1_(*x*) + *h*_*t*_(*x*)) of this cycle. This iteration finds the decision tree, and therefore, the sample loss is as small as possible.

Major step in this machine learning method is to minimize the loss function *L* through optimization. In the *t*-th iteration, the first *t* − 1 base learners are all fixed,

(1) $$\begin{array}{c} f_{t}\left(x\right)=f_{t-1}\left(x\right)+\rho_{t}h_{t}\left(x\right). \end{array}$$

Minimize loss function

(2) $$\begin{array}{c} L\left(f\right)=\overset{N}{\underset{i=1}{\Sigma }}L\left(y_{i},f_{t}\left(x_{i}\right)\right). \end{array}$$

The negative gradient of the loss function of the sample of the *t* wheel is expressed as

(3) $$\begin{array}{c} h_{t}\approx -\frac{\partial L\left(y_{i},f_{t-1}\left(x_{i}\right)\right)}{\partial f_{t-1}\left(x_{i}\right)}. \end{array}$$

Input cancer sample training set:

(4) $$\begin{array}{c} T=\left\{\left(x_{1},y_{1}\right),\left(x_{2},y_{2}\right),\cdots x_{N},y_{N}\right\}. \end{array}$$

*N*is the number of 7633 cancer samples, the maximum number of iterations is *T*, the loss function is *L*, and output maximum learner is *f*(*x*) = *f*_*T*_(*x*).

For a single tree *T*, the following formula for the importance of each feature *X*_l_ is used:

(5) $$\begin{array}{c} \Gamma_{l}^{2}\left(T\right)=\overset{Q-1}{\underset{t=1}{\Sigma }}{\overset{\wedge }{i}}^{2}I\left(v\left(t\right)=l\right), \end{array}$$

where *Q* is the number of leaf nodes, *Q*‐1 is the number of internal nodes, *X*_*v*(*t*)_ is the splitting characteristic associated with the internal node*t*where*t*is for the cancer type, and*l*is the number of features. For each internal node *t*, the feature *X*_*v*(*t*)_ is used to simulate and divide the feature space to obtain a square error reduction after splitting, that is, ${\overset{\wedge }{i}}^{2}$. Finally, the importance of feature *X*_l_ is summed up by the error reduction on all internal nodes. The more the total error is reduced, the more important this feature is. Because similar response values are in the same set, every node in the decision trees is a condition on a single gene. The more the total error decreases, the more important the feature becomes. For the integration of *M* trees, feature importance is the average of corresponding values of each tree.

Unlike GBDT, AdaBoost selects an exponential loss, while GBDT uses the classifying loss of function from the logistic loss *L*(*y*, *f*(*x*)) = log(1 + *e*^−2*yf*(*x*)^). We expected to minimize the loss of the function; therefore, we used the derivative of the function to find the minimum value of the function. After getting *f*_*T*_(*x*), we have to do the probability estimation by *P* = *P*(*y* = 1|*x*) = 1/(1 + *e*^−2*f*(*x*)^).

## 3. Results and Discussion

### 3.1. Workflow

The study process for identifying the tumor-of-origin was shown in Figure 1. Firstly, the expression profiles were downloaded from TCGA. A preprocess for the raw data was carried out before feature selection, which was performed by using the gradient boosting algorithm with 10-fold cross-validation. Then, final classification across 20 types of cancer was conducted by utilizing gradient boosting classifier, and the output of the model was displayed as an evaluation metric.

### 3.2. Data Preparation

From TCGA (Cancer Genome Atlas Research, 2008) data set, we downloaded expression profiles for 7713 RNA-seq samples covering 21 common cancers without metastasis [19]. Two samples were removed because of lack of clinical data. Then, we used RSEM to normalize these data.  Table 1 summarized these data and showed the information for tumor samples.

372 metastasis samples containing 352 cases with SKCM were originally included in the test data set. However, the metastatic cases that originated from SKCM are relatively higher than those from other cancers. In order to reduce impact on the results, SKCM data were removed during data analysis.

### 3.3. 400 Genes Were Selected for Future Prediction

20,501 genes across 7713 samples from the TCGA data set were included in the study. In order to reduce the model complexity, we performed feature selection. First, we ranked genes by importance scores calculated by gradient boosting algorithm, and the order was defined from high to low. We conducted a series of experiments, and the experimental results are shown in Figure 2. Based on the experimental results, we selected the feature number with highest accuracy. The top 400 gene features were extracted from each sample to construct a 7633 × 400 matrix [7]. This new matrix was the input for the classification of various cancers.

### 3.4. Classification

In the gene selection part, we got a 7633 × 400 matrix as the input matrix, and the corresponding gene expression profile of each sample was extracted. By using the GBDT method, we set n_estimators to 200. In fact, we also tested the estimator value from 100 to 300, and the results showed an upward trend followed downward trend and reached the maximum value at 200. Therefore, we finally chose 200 weak classifiers, which meant the number of decision trees was 200. The trained tree was used to select each cancer and returned the cancer which has been selected more times. We used the gene expression values as the training features to fit the cancer type as labels.

We adopted a 10-fold cross-validation in this study, which divided the data set into 10 subsets. Nine subsets were merged to a training set, and one subset was used as the test set. We repeated the algorithm ten times using the same gene features, and the average precision was 96.1%.

The confusion matrix is a standard format for precise evaluation, which is represented by an *M*∗*M* matrix. A confounding matrix can be used to judge the accuracy of the classifier classification and is presented in the form of a graph, so it is widely used to measure the success rate of classification. The confusion matrix is a summary of the predicted results of the classification problem. It can find errors in the classification model and understand the types of errors that are occurring [20, 21]. The confusion matrix of the classification using 400 genes shown in Figure 3 exhibited the sample number of a certain type of cancer that was classified into another type.

We also made a comparison with *K*-nearest neighbor (*K* = 5) [22], decision tree [23], AdaBoost [24], and support vector machine [25]. The results are shown in Figure 4. The results of *K*-nearest neighbor (*K* = 5) are closer to GBDT; GBDT is significantly higher than the other methods.

Table 2 showed correct and incorrect predictions of each type of cancer. For example, it is TCGA-BRCA but was predicted to be TCGA-LIHC or TCGA-BLCA, and it is TCGA-CESC but was identified to be TCGA-UCEC. As shown in Table 1, BRCA, LIHC, BLCA, CESC, and UCEC, respectively, represented breast invasive carcinoma, liver hepatocellular carcinoma, bladder urothelial carcinoma, cervical squamous cell and carcinoma endocervical adenocarcinoma, and uterine corpus endometrial carcinoma. Except for the above cases, the overall prediction accuracy was reaching 85%.

In order to verify the generalization and robustness of the approach, we also downloaded data sets from GEO for independent validation. The data sets covered 6 cancer types, including BRCA, LUAD, PAAD, PRAD, STAD, and THCA. And the overall accuracy rate from the gradient boosting classifier reached 83.5%.We also made a comparison with *K*-nearest neighbor (*K* = 5), decision tree, AdaBoost, and support vector machine. The results are shown in Figure 5. The results of *K*-nearest neighbor (*K* = 5) are closer to GBDT; GBDT is significantly higher than the other methods.

Biological validation of the optimal biomarker signature was done by GO enrichment analysis. The Gene Ontology (GO) Consortium was formed to address the limited interoperability of genomic databases due to lack of progress [26]. Figures 6 and 7 are the result of the GO enrichment analysis. The enrichment results showed that the genes were significantly enriched in maintenance and regulation of cell differentiation during morphogenesis of human organs and suborgan tissues, such as cell differentiation in kidney and prostate gland morphogenesis, reproductive system development, urogenital system development, epithelial tube morphogenesis, and mesenchymal cells. There are other genes involved in the hormone-mediated signaling pathway, cell proliferation, angiogenesis and apoptosis, and thyroid hormone regulation. Overall, the genes were enriched in negatively regulating organ morphogenesis, positively regulating cell differentiation during morphogenesis, and inducing cell apoptosis. Remarkably, some genes involved in organ- or tissue-specific development are more likely to be differentially expressed in tumors and normal tissues. The HOXB13 gene which belongs to the HOX superfamily was highly enriched in prostate adenocarcinoma. Increased expression from the HoxB13 is indicative of an invasive or metastatic status as well as increases cellular migration and/or mobility. The HoxB13 expression level could be a potential marker to evaluate clinical diagnosis as well as patient prognosis [27–32].

In Figures 8–11, we presented the results of 10 times 10-fold cross-validation. Precision refers to the proportion of the correct model prediction among all results that the model prediction is positive. Recall refers to the ratio of the number of correctly predicted positive samples to the total number of true positive samples, that is, how many positive samples can be correctly identified from these samples. Specificity, which is relative to recall, refers to the ratio of correctly predicted negative samples to the total number of true negative samples. In other words, how many negative samples can be correctly identified from these samples. The F1 score is equivalent to the harmonic average of precision and precision. If any number of the recall and precision decreases, the F1 score will decrease.

A heat map is a visualization method to analyze the distribution of experimental data, which directly reflected the expression of 400 characteristic genes in cancer species. As shown in Figure 12, the expression levels of the top 50 characteristic genes in the cancer species were relatively average, among which C19orf33, CRYAB, ACTG2, ACTA2, IGFBP2, CSRP1, RAB34, SMS, MAGOH, C21orf33, IDI1, TRIM27, ACTL6A, and ILVBL gained higher expression, while OR14A16, CRP, and INS had lower expression.

### 3.5. Discussion

The treatment of cancers with unknown primary origin is mainly empirical chemotherapy, but the prognosis of patients is generally poor. A clear diagnosis directly determines the surgical method and scope, as well as the drug regimen of physicians. Because the method in this paper is based on sequencing, this approach guides medication in patients who are sequenced. For patients who are not sequenced, the next step of diagnosis and treatment should be determined according to the guidance of doctors. The diagnostic techniques primarily include comprehensive evaluation, imaging examination, pathological analysis, immunohistochemistry (IHC) panels, and genetic testing, but the treatment is less effective. The method proposed in this paper can be used to identify tumor tissue of origin, so as to provide doctors with help and appropriate drugs according to this.

We used GBDT to predict the tissue origin of the metastatic samples. GBDT can flexibly handle all kinds of data, including continuous value and discrete value. GBDT uses some robust loss functions and is relatively robust to outliers such as the Huber loss function and the quantile loss function. Because of the dependence among weak learners, it is difficult to carry out parallel training. Therefore, if the program runs too slowly with a large amount of data, it can achieve partial parallelism by adding self-sampling SGBT. The training data in this experiment was not parallel to the training data. Therefore, the results of this study might be influenced by the training method.

It was demonstrated that GBDT is a powerful method of ensemble learning. Breast cancer has a high mortality rate and is the most common cancer among women worldwide. Because of the high mortality rate of breast cancer patients, the most urgent need is to find appropriate biomarkers to determine the prognosis of breast cancer, especially BRCA (invasive breast cancer) [33]. Because basal cells like breast cancer, serous ovarian cancer, and lung squamous carcinoma have a high mRNA expression, tumors from different organs may have the same oncogenic driver events [34, 35]. Endometrial cancer is a common type of endometrial cancer, and the increase of age brings an increase in the incidence of UCES. Therefore, women aged between 45 and 65 are more likely to develop endometrial cancer than women of other ages [36, 37]. Cervical neoplasm is histologically classified like squamous cell carcinoma, adenocarcinoma, and so on. Squamous cell carcinoma accounts for 85-90% of the total cervical cancer, and adenocarcinoma accounts for the rest [38].

Neither the TCGA test set nor GEO's independent test set was 100 percent accurate because a small percentage of cancers were misdiagnosed. The main reason for this error is that the two cancer species have similar characteristics and are easy to misjudge during classification, which is a key point that can be improved in the future.

Since this study was researched on gene expression profiles, it is easy to make an error prediction if the gene expressions of samples are similar. Therefore, the next step was to address this problem by increasing the sample number in types of cancer.

## 4. Conclusions

In conclusion, we applied a gradient boosting classifier to identify 20 tumor types based on expression profiles with a high accuracy, which might assist the pathologists in the diagnosis of cancers of unknown primary origins. Subsequent work has been to improve accuracy by increasing the number of samples of cancer types and improving methods.

## Figures and Tables

**Figure 1:** Flow chart of identification of tumor tissue origin.

**Figure 2:** Accuracies of different numbers of genes with cross-validation.

**Figure 3:** Confusion matrix of the classification using 400 genes.

**Figure 4:** Accuracies of five different algorithms based on TCGA.

**Figure 5:** Accuracies of five different algorithms based on GEO.

**Figure 6:** GO enrichment analysis about pathway.

**Figure 7:** Specific cluster.

**Figure 8:** F1 score for each cancer.

**Figure 9:** Precision for each cancer.

**Figure 10:** Recall for each cancer.

**Figure 11:** Specificity for each cancer.

**Figure 12:** Average gene expression for each cancer.

**Algorithm 1:** Algorithm 1: Gradient boosting.

**Table 1:** The disease name and sample number in TCGA data.

Disease	Code	Tumor samples	Percentage
Bladder urothelial carcinoma	BLCA	301	3.9025%
Breast invasive carcinoma	BRCA	1056	13.6912%
Cervical squamous cell carcinoma and endocervical adenocarcinoma	CESC	258	3.3450%
Colon adenocarcinoma	COAD	451	5.8473%
Glioblastoma multiforme	GBM	153	1.9837%
Head and neck squamous cell carcinoma	HNSC	480	6.2233%
Kidney renal clear cell carcinoma	KIRC	526	6.8197%
Kidney renal papillary cell carcinoma	KIRP	222	2.8783%
Acute myeloid leukemia	LAML	173	2.2430%
Brain lower grade glioma	LGG	439	5.6917%
Liver hepatocellular carcinoma	LIHC	294	3.8117%
Lung adenocarcinoma	LUAD	486	6.3011%
Lung squamous cell carcinoma	LUSC	428	5.5491%
Ovarian serous cystadenocarcinoma	OV	261	3.3839%
Pancreatic adenocarcinoma	PAAD	142	1.8410%
Prostate adenocarcinoma	PRAD	379	4.9138%
Rectum adenocarcinoma	READ	153	1.9837%
Skin cutaneous melanoma	SKCM	80	1.0372%
Stomach adenocarcinoma	STAD	415	5.3805%
Thyroid carcinoma	THCA	500	6.4826%
Uterine corpus endometrial carcinoma	UCEC	516	6.6900%
Total		7713	

**Table 2:** Correctly and incorrectly predicting the type of cancer.

Predicted_label	True_label	Matched_label
TCGA-BRCA	TCGA-BRCA	1
TCGA-BRCA	TCGA-BRCA	1
TCGA-LIHC	TCGA-BRCA	0
TCGA-BLCA	TCGA-BRCA	0
TCGA-BRCA	TCGA-BRCA	1
TCGA-BRCA	TCGA-BRCA	1
TCGA-BRCA	TCGA-BRCA	1
TCGA-UCEC	TCGA-CESC	0
TCGA-CESC	TCGA-CESC	1
TCGA-COAD	TCGA-COAD	1
TCGA-HNSC	TCGA-HNSC	1
TCGA-HNSC	TCGA-HNSC	1
TCGA-THCA	TCGA-THCA	1
TCGA-THCA	TCGA-THCA	1
TCGA-THCA	TCGA-THCA	1
TCGA-THCA	TCGA-THCA	1
TCGA-THCA	TCGA-THCA	1
TCGA-THCA	TCGA-THCA	1
TCGA-THCA	TCGA-THCA	1
TCGA-THCA	TCGA-THCA	1

## Data Availability

The Cancer Genome Atlas (TCGA) RNA-seq and array data include 20,501 genes from the ICGC Data Portal (https://dcc.icgc.org/releases/release_26/) download. An independent data set was also downloaded from the Gene Expression Omnibus (GEO). These samples belong to GSE8352, GSE8734, GSE11107, GSE11132, GSE4895, GSE6491, GSE7966, GSE7766, and GSE11843.

## Supplementary Materials

Supplementary Materials The file in the name of “The Selection of 400 Genes.docx” contains the names of the 400 genes selected.
